# Physiological Stress Elicits Impaired Left Ventricular Function in Preterm-Born Adults

**DOI:** 10.1016/j.jacc.2018.01.046

**Published:** 2018-03-27

**Authors:** Odaro J. Huckstep, Wilby Williamson, Fernando Telles, Holger Burchert, Mariane Bertagnolli, Charlotte Herdman, Linda Arnold, Robert Smillie, Afifah Mohamed, Henry Boardman, Kenny McCormick, Stefan Neubauer, Paul Leeson, Adam J. Lewandowski

**Affiliations:** a Oxford Cardiovascular Clinical Research Facility, Division of Cardiovascular Medicine, Radcliffe Department of Medicine, University of Oxford, Oxford, United Kingdom; b Department of Paediatrics, University of Oxford, Oxford, United Kingdom; c Oxford Centre for Clinical Magnetic Resonance Research, Division of Cardiovascular Medicine, Radcliffe Department of Medicine, University of Oxford, Oxford, United Kingdom

**Keywords:** cardiac function, echocardiography, ejection fraction, heart failure, myocardial reserve, premature, preterm, BSA, body surface area, CI, cardiac index, CMR, cardiovascular magnetic resonance, COR, cardiac output reserve, CPET, cardiopulmonary exercise test, EDV, end-diastolic volume, EF, ejection fraction, ESV, end-systolic volume, LV, left ventricular

## Abstract

**Background:**

Experimental and clinical studies show that prematurity leads to altered left ventricular (LV) structure and function with preserved resting LV ejection fraction (EF). Large-scale epidemiological data now links prematurity to increased early heart failure risk.

**Objectives:**

The authors performed echocardiographic imaging at prescribed exercise intensities to determine whether preterm-born adults have impaired LV functional response to physical exercise.

**Methods:**

We recruited 101 normotensive young adults born preterm (n = 47; mean gestational age 32.8 ± 3.2 weeks) and term (n = 54) for detailed cardiovascular phenotyping. Full clinical resting and exercise stress echocardiograms were performed, with apical 4-chamber views collected while exercising at 40%, 60%, and 80% of peak exercise capacity, determined by maximal cardiopulmonary exercise testing.

**Results:**

Preterm-born individuals had greater LV mass (p = 0.015) with lower peak systolic longitudinal strain (p = 0.038) and similar EF to term-born control subjects at rest (p = 0.62). However, by 60% exercise intensity, EF was 6.7% lower in preterm subjects (71.9 ± 8.7% vs 78.6 ± 5.4%; p = 0.004) and further declined to 7.3% below the term-born group at 80% exercise intensity (69.8 ± 6.4% vs 77.1 ± 6.3%; p = 0.004). Submaximal cardiac output reserve was 56% lower in preterm-born subjects versus term-born control subjects at 40% of peak exercise capacity (729 ± 1,162 ml/min/m^2^ vs. 1,669 ± 937 ml/min/m^2^; p = 0.021). LV length and resting peak systolic longitudinal strain predicted EF increase from rest to 60% exercise intensity in the preterm group (r = 0.68, p = 0.009 and r = 0.56, p = 0.031, respectively).

**Conclusions:**

Preterm-born young adults had impaired LV response to physiological stress when subjected to physical exercise, which suggested a reduced myocardial functional reserve that might help explain their increased risk of early heart failure. (Young Adult Cardiovascular Health sTudy [YACHT]; NCT02103231)

Preterm birth rates range from 5% to 18% worldwide (1). The population of adults born preterm has risen sharply in recent decades because modern perinatal care often achieves 95% survival rates (2). Multiple studies have described a distinct preterm cardiovascular phenotype, including altered cardiac structure and function 3, 4, 5 and impaired exercise capacity (6), as well as increased risk for hypertensive disorders and stroke (7). However, as the modern cohorts of preterm-born survivors now approach middle age, the long-term epidemiological consequences of prematurity remain largely unknown. A recently reported study of >2.6 million individuals born between 1987 and 2012 identified preterm birth as a novel risk factor for incident heart failure in childhood and adolescence (8), emphasizing the importance of research into the underlying mechanisms responsible for increased risk in this population.

Acute cardiac insufficiency is uncommon in young adults (9) and a previous cardiovascular magnetic resonance (CMR) study confirmed that preterm-born young adults maintain a fully preserved resting left ventricular (LV) ejection fraction (EF) despite significant functional and anatomical LV remodeling (4). Stress echocardiography is a powerful tool used to unmask underlying cardiac dysfunction that is well-compensated at rest by assessing the cardiac response to physiological stressors such as exercise (10). Because those born preterm have well compensated resting LV function despite significant structural modifications and moderate changes in myocardial deformation at rest (4), investigating cardiac functional responses to physiological stress is essential to more fully understand the impact of being born preterm on LV function (10). We therefore used 2-dimensional echocardiography to test the hypothesis that the LV of preterm-born young adults has reduced myocardial reserve that results in functional impairment in response to the physiological stressor of physical exercise.

## Methods

### Study design

We completed YACHT (Young Adult Cardiovascular Health sTudy), an observational, case−control study to investigate cardiovascular structure, function, and physiological stress response in preterm and term-born young adults. Participants age 18 to 40 years completed a detailed multimodal set of study measures, including 24-h ambulatory blood pressure monitoring, cardiopulmonary exercise testing, and cardiac imaging. Ethical approval for YACHT was granted by the South Central Berkshire Research Ethics Committee (14/SC/0275). Study registration was completed via ClinicalTrials.gov (NCT02103231).

### Study population

A total of 149 participants were recruited into YACHT through open recruitment in the local Oxford community using posters, mailed invitations from the John Radcliffe Hospital birth registries, word of mouth, patient invitation through the John Radcliffe Hospital Specialist Hypertension Clinic, and invitations to previous study participants who had indicated interest in future study participation. In total, 48 participants were excluded from this analysis to prevent confounding: 32 diagnosed hypertensive participants recruited through the John Radcliffe Hospital Hypertension Clinic, and 16 additional participants with awake ambulatory blood pressure measures in the hypertensive range. Therefore, 101 nonhypertensive young adult participants (47 preterm-born, 54 term-born) who met the following criteria were recruited and included in this analysis: 1) aged 18 to 40 years; 2) body mass index <40 kg/m^2^; 3) awake ambulatory blood pressure <135/85 mm Hg; and 4) verified birth history (preterm or term-born). Exclusion criteria included: 1) unwilling or unable to give informed consent; 2) pregnant or lactating; 3) history of acute cardiac or cerebrovascular event; 4) diagnosis with a disease or disorder that could influence study participation or outcome measures; 5) hypertension diagnosis; and 6) treatment with antihypertensive medication. Participants were assessed with a wide range of measures to achieve deep cardiovascular phenotyping, including clinic and 24-h ambulatory blood pressure, biochemistry, anthropometry, cardiopulmonary exercise testing, vascular stiffness, multiorgan magnetic resonance imaging, as well as a full clinical resting echocardiogram and stress echocardiogram using apical 4-chamber views while exercising at 40%, 60%, and 80% of peak exercise capacity. Cohort characteristics are provided in Table 1.

**Table 1:** Cohort Characteristics

	Preterm-Born Adults (n = 47)	Term-Born Adults (n = 54)	p Value
Demographics and anthropometrics			
Age, yrs	22.7 ± 3.0	23.6 ± 3.8	0.239
Male	14 (30.0)	26 (48.0)	0.061
Height, cm	167 ± 9	175 ± 10	**<0.001**
Weight, kg	65.3 ± 13.5	70.0 ± 13.0	0.299
Body surface area, m^2^	1.73 ± 0.19	1.84 ± 0.21	**0.010**
BMI, kg/m^2^	23.3 ± 4.5	22.7 ± 2.7	0.401
Birth weight, g	1,916 ± 806	3,390 ± 424	**<0.001**
Birth weight, g	595–3203	2640–4536	**<0.001**
Gestational age, weeks	32.80 ± 3.22	39.50 ± 1.37	**<0.001**
Gestational age, weeks	23–36	38–42	**<0.001**
Gestational hypertension	8 (17.0)	0 (0.0)	**0.002**
Small for gestational age	2 (4.3)	0 (0.0)	0.214
Biochemistry			
Total cholesterol, mmol/l	4.72 ± 0.65	4.18 ± 0.77	**0.001**
HDL, mmol/l	1.49 ± 0.31	1.47 ± 0.26	0.953
LDL, mmol/l	2.80 ± 0.71	2.32 ± 0.60	**0.001**
Triglycerides, mmol/l	1.12 ± 0.66	0.87 ± 0.36	**0.031**
High-sensitivity CRP, mg/l	1.57 ± 2.42	1.14 ± 1.96	0.412
Glucose, mmol/l	5.02 ± 0.41	4.82 ± 0.51	**0.030**
Insulin, pmol/l	51.1 ± 29.0	35.8 ± 29.4	**0.012**
Insulin resistance	0.96 ± 0.54	0.68 ± 0.59	**0.020**
Brachial blood pressure, mm Hg			
Resting systolic	119 ± 9	115 ± 8	**0.014**
Resting diastolic	70 ± 8	66 ± 5	**0.014**
Awake average ambulatory systolic	119 ± 6	119 ± 8	0.610
Awake average ambulatory diastolic	71 ± 5	69 ± 5	0.058

Values are mean ± SD, n (%), or range. Insulin resistance was calculated using the Homeostatis Model Assessment calculator. p values were adjusted for sex. **Bold** p values are statistically significant (p < 0.05).

BMI = body mass index; CRP = C-reactive protein; HDL = high-density lipoprotein; LDL = low-density lipoprotein.

### Study visit

#### Overview

Participants were instructed to fast overnight for 12 h but encouraged to drink water to remain hydrated before attending a study visit at the University of Oxford Centre for Clinical Magnetic Resonance Research and Oxford Cardiovascular Clinical Research Facility in the John Radcliffe Hospital (Oxford, United Kingdom). All measurements were completed by trained study investigators.

#### Anthropometry

Using an integrated height and weight measurement station (Seca, Birmingham, United Kingdom), height was measured to the nearest centimeter and weight measured to the nearest 0.1 kg with footwear removed and participants wearing light clothing. Manual waist circumference was measured 2 cm above the iliac crest, and manual hip measurements were taken at the point of widest overall girth near the level of the greater trochanter of the femur or mid-buttock.

#### Blood pressure

After a 5-min acclimation period, 3 resting peripheral blood pressure measurements were recorded using a digital blood pressure monitor (GE Dinamap V100, GE Healthcare, Chalfont St. Giles, United Kingdom) on the left arm with the last 2 readings averaged and subsequently analyzed. Twenty-four-hour ambulatory blood pressure monitoring was initiated at the end of the study visit using oscillometric, ambulatory devices (TM-2430, A&D Instruments, Abingdon, United Kingdom). Correct cuff size was chosen based on arm circumference. Subjects were instructed to remain still during measurements. Measurements were automatically taken every 30 min during daytime and then hourly from 11:00 pm to 7:00 am. Subjects completed a diary documenting hours asleep and awake.

#### Blood sampling

All blood samples were collected from the antecubital fossa by venipuncture or indwelling venous catheter. After collecting fasting, at-rest blood samples, participants were provided a standardized snack of 2 cereal bars. Samples were centrifuged within 15 min of collection. Separated plasma and serum were then pipetted and stored at −80°C for future analysis. Fasting blood biochemistry was measured at the Oxford John Radcliffe Hospital Biochemistry Laboratory using routine validated assays with clinical level quality controls. Insulin resistance was calculated using the homeostasis model assessment calculator (11).

#### Resting echocardiography

Resting transthoracic echocardiography was performed in the left lateral decubitus position using a commercially available Philips iE33 or Philips EPIQ 7C cardiology ultrasound machine. British Society of Echocardiography guidelines were followed for collection of a standard clinical imaging data set to quantify LV dimensions and systolic and diastolic function, as well as review valvular function (12).

#### Cardiopulmonary exercise test

Participants completed a peak cardiopulmonary exercise test (CPET) on a seated stationary cycle ergometer (Ergoline GmbH, Bitz, Germany) using a validated incremental protocol, with respiratory gases collected and measured (Metalyzer 3B, Cortex Biophysik, Leipzig, Germany). Heart rate was recorded using continuous electrocardiographic monitoring, whereas the rate of perceived exertion was recorded every 2 min, and blood pressure was recorded every 4 min using a manual mercury sphygmomanometer (Accoson Freestyle, Essex, United Kingdom). Participants were instructed to maintain a rate of 60 rpm during the test, which began with 1 quiescent min of resting measurements followed by a 2-min warmup with a 20 W workload. After the warmup period, workload increased to 35 W. To normalize test duration to approximately 8 to 12 min, participants who reported higher activity or fitness levels had their workload increased to 75 W after the warmup period. Workload was then incremented by 15 W each min, and participants cycled continuously until exhaustion prevented them from maintaining at least 50 rpm. Participants then completed a 2-min cool down period at 35 W and the rpm of their preference. Following the cool down period, participants were transferred to a reclined treatment bed for post-exercise venous blood sampling.

#### Stress echocardiography

After completing CPET testing, participants had a 30-min recovery period during which they were offered water and an additional cereal bar. Submaximal exercise stress echocardiography was then performed on study subjects for 3 min at 40%, 60%, and 80% of their peak exercise wattage achieved during CPET testing. After participants exercised at each prescribed workload for 2 min, and steady-state heart rate was verified, apical 4-chamber views oriented for optimal imaging of the LV and pulsed wave Doppler imaging of mitral inflow were collected at each stage using either a Philips iE33 or Philips EPIQ 7C cardiology ultrasound machine (Philips Healthcare, Surrey, United Kingdom). Participants were given a 3-min rest period between each stage. Off-line image analysis was only performed on images in which heart rate was within 5% of maximum achieved steady-state heart rate for a given stage.

### Data processing

#### Echocardiographic analysis

Echocardiographic analysis was completed off-line in accordance with standard guidelines from the European Association of Echocardiography and the American Society of Echocardiography 13, 14, 15 by a single blinded investigator to minimize bias and intraobserver variation. The Philips Xcelera 3.3 (Philips Healthcare Informatics, Belfast, United Kingdom) and TomTec Image Arena 4.6 software suites (TomTec, Chicago, Illinois) were used for image analysis. End-diastole was set at the point of mitral valve closure, and end-systole was set at the point of minimum LV cavity size. LV endocardial borders were manually contoured at end-diastole and end-systole to allow calculation of end-diastolic volume (EDV) and end-systolic volume (ESV). Resting EFs were then calculated via the biplane modified Simpson’s method using apical 4-chamber and apical 2-chamber views, whereas submaximal exercise EFs were calculated by the single-plane modified Simpson’s method using apical 4-chamber views. Ten imaging data sets were randomly selected and re-evaluated for intraobserver and interobserver variability. Intraclass correlation coefficients for LV mass, EF, stroke volume, EDV, longitudinal strain, longitudinal systolic strain rate, and longitudinal diastolic strain rate for intraobserver and interobserver variability yielded: 0.99 and 0.96; 0.89 and 0.85; 0.92 and 0.88; 0.94 and 0.91; 0.93 and 0.86; 0.86 and 0.81; and 0.95 and 0.90, respectively.

#### Submaximal cardiac output reserve calculation

Submaximal cardiac output reserve was calculated similarly to previous studies (16). Briefly, cardiac output indexed to body surface area (BSA) was calculated at rest (cardiac index [CI_rest_]) and also at 40%, 60%, and 80% exercise intensity (CI_40_, CI_60,_ CI_80_) by multiplying heart rate in beats per min by stroke volume indexed to BSA, measured using echocardiography. Submaximal cardiac output reserve (COR) values at 40%, 60%, and 80% exercise intensity (COR_40_, COR_60,_ COR_80_) were then calculated by subtracting CI_rest_ from the calculated CI at each exercise intensity (CI_40_, CI_60_, CI_80_). The units for both CI and COR are ml/min/m^2^. The submaximal COR equations are as follows: COR_40_ = CI_40_ − CI_rest_; COR_60_ = CI_60_ − CI_rest_; and COR_80_ = CI_80_ − CI_rest_.

### Statistical analysis

Statistical analysis was performed using SPSS (version 23, IBM, Armonk, New York). Shapiro-Wilk testing and visual inspection were used to assess whether variables were normally distributed. Direct between-group comparisons were performed using independent-samples Student’s *t*-tests for normally distributed data and Mann-Whitney and Kruskal-Wallis tests for non-normally distributed data. Linear regression modeling was completed using forced entry with missing data excluded pairwise. Standardized regression coefficients (β) are presented for multivariate linear regressions. Pearson correlations (r) were used for bivariate correlations. The study was powered at 80%, and p = 0.05 to detect a 0.77 SD difference between groups for LV exercise echocardiographic measures. Where appropriate, comparisons between term-born and preterm-born adults were adjusted for sex by multivariate linear regression modeling to account for differing sex distributions between groups. This includes demographic, anthropometric, biochemistry, blood pressure, and LV echocardiography measures. Values of p < 0.05 were considered statistically significant.

## Results

### Clinical characteristics

The gestational age of the preterm group was lower than the term-born control subjects (32.8 ± 3.22 weeks vs. 39.5 ± 1.37 weeks; p < 0.001). The gestational age range for the preterm cohort was 23 to 36 weeks. However, 80.9% (n = 38 of 47) were born moderate to late pre-term (32 to 36 weeks), 10.6% (n = 5 of 47) were born very preterm (28 to 31 weeks), and 8.5% (n = 4 of 47) were born extremely preterm (<28 weeks). Height and BSA were lower in the preterm group. There were no differences in body mass index or age, but between-group sex distribution approached significance, with a 30% male preterm group versus a 48% male term-born group (p = 0.061). Both groups had similar average awake ambulatory systolic and diastolic pressures; however, the preterm group had higher resting systolic (119 ± 9 mm Hg vs. 115 ± 8 mm Hg; p = 0.014) and resting diastolic (70 ± 8 mm Hg vs. 66 ± 5 mm Hg; p = 0.014) clinic blood pressure readings (Table 1).

### Resting echocardiography

#### Altered LV structure in preterm-born adults

Two-dimensional echocardiography of the LV showed the preterm group had a greater LV mass indexed to BSA (69.1 ± 13.5 g/m^2^ vs. 63.7 ± 14.7 g/m^2^; p = 0.015) and a greater LV mass indexed to EDV (1.54 ± 0.33 g/ml vs. 1.22 ± 0.27 g/ml; p < 0.001). Additional adjustment for systolic blood pressure did not affect these between-group differences for LV mass indexed to BSA (p = 0.022) and LV mass indexed to EDV (p < 0.001). Those born preterm had smaller LV internal cavity diameters at end-diastole (4.50 ± 0.41 cm vs. 4.82 ± 0.51 cm; p = 0.007), with lower EDV indexed to BSA (46.4 ± 9.7 ml/m^2^ vs 52.5 ± 12.7 ml/m^2^; p = 0.037) (Table 2).

**Table 2:** Left Ventricular Resting Echocardiography

	Preterm-Born Adults (n = 47)	Term-Born Adults (n = 54)	p Value
Structure			
Mass index, g/m^2^	69.1 ± 13.5	63.7 ± 14.7	**0.015**
Mass/EDV, g/ml	1.54 ± 0.33	1.22 ± 0.27	**<0.001**
End-diastolic diameter, cm	4.50 ± 0.41	4.82 ± 0.51	**0.007**
End-diastolic length, cm	7.75 ± 0.81	8.15 ± 0.97	0.169
EDV, ml	80.4 ± 21.5	97.5 ± 28.7	**0.010**
EDV/BSA, ml/m^2^	46.4 ± 9.7	52.5 ± 12.7	**0.018**
ESV/BSA, ml/m^2^	16.9 ± 4.7	20.3 ± 6.4	**0.037**
Function			
Heart rate, beats/min	68.8 ± 24.4	58.8 ± 16.3	**0.023**
Ejection fraction, %	63.1 ± 5.4	63.4 ± 4.7	0.624
Stroke index, ml/m^2^	29.6 ± 6.4	32.2 ± 7.8	0.173
Fractional area change, %	48.9 ± 5.6	49.4 ± 5.7	0.396
Cardiac output, l/min	3.78 ± 0.89	3.62 ± 0.56	0.224
IVRT, s	0.085 ± 0.019	0.088 ± 0.022	0.517
E/A ratio	1.52 ± 0.38	1.75 ± 0.42	**0.013**
E, cm/s	82.1 ± 13.1	86.1 ± 15.5	0.125
A, cm/s	56.3 ± 12.5	51.0 ± 12.5	0.096
E-wave deceleration time, ms	0.23 ± 0.05	0.23 ± 0.05	0.723
Diastolic filling time, s	0.46 ± 0.13	0.61 ± 0.15	**<0.001**
E-VTI, cm	12.8 ± 2.5	13.6 ± 2.1	0.163
A-VTI, cm	4.93 ± 1.18	4.38 ± 1.12	**0.035**
E-VTI/A-VTI	2.77 ± 0.95	3.22 ± 0.74	**0.021**
2-Dimensional peak strain			
Longitudinal			
Systolic strain, %	−19.7 ± 2.7	−20.6 ± 3.0	**0.038**
Systolic strain rate, %/s	−1.17 ± 0.19	−1.11 ± 0.37	0.590
Diastolic strain rate, %/s	1.62 ± 0.48	1.77 ± 0.58	0.082
Radial			
Systolic strain, %	49.2 ± 17.5	45.1 ± 12.7	0.285
Systolic strain rate, %/s	2.50 ± 1.03	2.36 ± 0.73	0.585
Diastolic strain rate, %/s	−3.11 ± 1.41	−2.88 ± 1.15	0.555
Circumferential			
Systolic strain, %	−26.6 ± 4.0	−27.0 ± 3.8	0.321
Systolic strain rate, %/s	−1.67 ± 0.30	−1.57 ± 0.28	0.156
Diastolic strain rate, %/s	2.26 ± 0.70	2.14 ± 0.58	0.706

Values are mean ± SD. p values were adjusted for sex. **Bold** p values are statistically significant (p < 0.05).

A = peak atrial systolic velocity of transmitral flow; BSA = body surface area; E = peak early diastolic velocity of transmitral flow; EDV = end-diastolic volume; IVRT = isovolumetric relaxation time; VTI = velocity−time integral.

#### Altered resting LV function with preserved EF in preterm-born adults

The preterm group had a higher resting heart rate (68.8 ± 24.4 beats/min vs. 58.8 ± 16.3 beats/min; p = 0.023) but a similar resting EF compared with those born at-term (63.1 ± 5.4% vs. 63.4 ± 4.7%; p = 0.62). However, the preterm group had a lower E-to-A ratio (1.52 ± 0.38 vs. 1.75 ± 0.42; p = 0.013), A velocity−time integral (4.93 ± 1.18 cm vs. 4.38 ± 1.12 cm; p = 0.035), as well as an E-to-A velocity−time integral (2.77 ± 0.95 cm vs. 4.38 ± 0.74 cm; p = 0.021). Peak systolic longitudinal strain was also lower in the preterm group at rest (−19.7 ± 2.7% vs. −20.6 ± 3.0%; p = 0.038) (Table 2).

### Cardiopulmonary exercise testing

#### Peak respiratory exchange ratio

The preterm and term-born groups both achieved the same respiratory exchange ratio at peak exercise intensity (1.19 ± 0.064 vs. 1.19 ± 0.064; p = 0.738).

### Exercise stress echocardiography

#### Impaired systolic response to exercise in preterm-born adults

LV function was not significantly different between groups at 40% of peak exercise intensity (EF: 75.6 ± 8.5% vs. 79.0 ± 5.2%; p = 0.115; peak systolic longitudinal strain: −21.3 ± 3.1% vs. −22.7 ± 2.7%; p = 0.103). However, at 60% exercise intensity, the EF of the preterm-born group dropped to 6.7% below the control subjects (71.9 ± 8.7% vs. 78.6 ± 5.4%; p = 0.004), with lower peak systolic longitudinal strain in the preterm group as well (−19.3 ± 2.5% vs. −21.6 ± 3.3%; p = 0.004). In addition, within the preterm-born group, there was a statistically significant 3.7% decline in EF when going from 40% to 60% exercise intensity (p = 0.039). EF remained lower in the preterm group compared with the term group at 80% exercise intensity (69.8 ± 6.4% vs. 77.1 ± 6.3%; p = 0.004). Stress echocardiography data are presented in Table 3, and EF from rest through all stages of exercise are presented in the Central Illustration. Comparisons between preterm-born and term-born individuals for EF at 40%, 60%, and 80% exercise intensity were repeated, adjusting for both sex and systolic blood pressure. EF at 40% exercise intensity did not differ between preterm-born and term-born adults (p = 0.387), but was significantly lower in preterm–born adults at 60% (p = 0.017) and 80% (p = 0.016).

**Central Illustration:** Left Ventricular Ejection Fraction With Increasing Exercise Intensity in Preterm-Born Versus Term-Born Young Adults Preterm-born young adults **(orange)** had a lower ejection fraction (EF) than term-born young adults **(blue)** at 60% and 80% of peak exercise intensity (71.9 ± 8.7% vs. 78.6 ± 5.4% and 69.8 ± 6.4% vs. 77.1 ± 6.3%, respectively; p < 0.005). In the preterm group, EF at 60% and 80% exercise intensity were both significantly lower than the within-group EF at 40% intensity (3.7% and 5.8% lower, respectively; p < 0.05). This declining EF with increasing exercise intensity was not observed in term-born control subjects. **Error bars** represent SEM. *Significantly lower EF than that in the term-born group (p < 0.005). †Significantly lower than the within-group EF at 40% (p < 0.05).

**Table 3:** Left Ventricular Exercise Echocardiography

	Preterm-Born Adults (n = 21)	Term-Born Adults (n = 37)	p Value
40% Exercise load			
Ejection fraction, %	75.6 ± 8.5	79.0 ± 5.2	0.115
Stroke volume index, ml/m^2^	21.4 ± 8.8	26.9 ± 7.6	0.104
EDV/BSA, ml/m^2^	27.6 ± 10.4	33.6 ± 10.0	0.760
ESV/BSA, ml/m^2^	6.68 ± 2.79	7.40 ± 3.34	0.147
Peak systolic longitudinal strain, %	−21.3 ± 3.1	−22.7 ± 2.7	0.103
60% Exercise load			
Ejection fraction, %	71.9 ± 8.7	78.6 ± 5.4	**0.004**
Stroke volume index, ml/m^2^	21.5 ± 10.6	25.6 ± 6.8	0.218
EDV/BSA, ml/m^2^	29.2 ± 11.5	32.8 ± 9.5	0.500
ESV/BSA, ml/m^2^	7.61 ± 2.27	7.20 ± 3.42	0.430
Peak systolic longitudinal strain, %	−19.3 ± 2.5	−21.6 ± 3.3	**0.004**
80% Exercise load			
Ejection fraction, %	69.8 ± 6.4	77.1 ± 6.3	**0.004**
Stroke volume index, ml/m^2^	19.9 ± 7.6	25.1 ± 6.9	0.094
EDV/BSA, ml/m^2^	28.1 ± 9.7	32.6 ± 8.7	0.154
ESV/BSA, ml/m^2^	8.24 ± 2.60	7.52 ± 3.12	0.420
Peak systolic longitudinal strain, %	−20.2 ± 2.9	−20.1 ± 2.4	0.592

Values are mean ± SD. p values were adjusted for sex. **Bold** p values are statistically significant (p < 0.05).

ESV = end-systolic volume; other abbreviation as in Table 2.

#### Reduced submaximal cardiac output reserve in preterm-born adults

Between-group comparison at 40% exercise intensity showed the preterm–born cohort had a 56% lower submaximal COR than that in term-born participants (729 ± 1,162 ml/min/m^2^ vs. 1,669 ± 937 ml/min/m^2^; p = 0.021). Mean submaximal CORs at 60% and 80% intensity were lower in the preterm-born group (41% and 45% lower, respectively) but were not statistically significant (p = 0.057 and p = 0.071, respectively) (Figure 1).

**Figure 1:** Submaximal Exercise Cardiac Output Reserve With Increasing Exercise Intensity in Preterm Versus Term-Born Young Adults Submaximal cardiac output reserve values at 40%, 60%, and 80% exercise intensity were calculated by subtracting resting cardiac index from the cardiac index at each exercise intensity level. Submaximal exercise cardiac output reserve at 40% of peak exercise intensity was 56% lower in the preterm-born group versus term-born control subjects (p = 0.021). **Error bars** represent SEM. **Bold** p values are statistically significant (p < 0.05).

#### Predictors of impaired systolic exercise response in preterm-born adults

With increasing workload from rest to 60% exercise intensity, the preterm-born group increased their EF by 8.1% compared with 15.2% in the term-born group (p = 0.039). To identify cardiac morphological predictors of this impaired systolic response to exercise, we selected resting structural and functional measures known to be modified in the preterm cardiac phenotype and performed correlation analyses of these parameters against the change in EF from rest to 60% exercise load (Table 4). Bivariate correlation showed that LV length and peak systolic longitudinal strain correlated to acute exercise-induced EF gains in the preterm group but not in term-born controls. However, in a multivariate model including both LV length and peak systolic longitudinal strain, LV length remained the only significant predictor of exercise systolic response in the preterm-born group (β = 0.51, p = 0.036). A linear regression plot of LV length versus EF change from rest to 60% exercise load in the preterm-born group is presented in Figure 2A (r^2^ = 0.46; p < 0.01), whereas the same values for the term-born group are plotted in Figure 2B and show no significant relationship (r^2^ = 0.02, p = 0.46). Gestational age was also related to LV length and exercise systolic response in bivariate correlations in the preterm group (r = 0.29, p = 0.059 and r = 0.67, p = 0.011), and therefore, an additional multivariate model was performed to explore the independent relationship with exercise systolic response. In this model, LV length and gestational age were included as independent variables, as was systolic blood pressure due to its potential confounding effect on the EF change from rest to 60% exercise intensity. Only LV length (β = 0.53, p = 0.016) and gestational age (β = 0.47, p = 0.027) remained as independent predictors of exercise systolic response in the preterm-born adults.

**Figure 2:** Relationship Between Left Ventricular Length and Change in Ejection Fraction When Going From Rest to 60% Exercise Intensity in Preterm-Born Versus Term-Born Young Adults **(A)** In preterm-born adults, greater left ventricular (LV) length was strongly correlated with increasing ejection fraction (EF) when going from rest to 60% exercise intensity (p < 0.01). **(B)** In term-born adults, LV length was not correlated with a change in EF when going from rest to 60% exercise intensity (p = 0.46).

**Table 4:** Predictors of Ejection Fraction Increase at 60% Exercise Load

	Preterm-Born Adults (n = 21)				Term-Born Adults (n = 37)			
	*m*	*b*	*r*	p Value	*m*	*b*	*r*	p Value
LV geometry								
End-diastolic internal diameter	7.15	−22.0	0.33	0.232	−1.39	23.0	−0.09	0.630
EDV/BSA	0.47	−11.4	0.51	0.052	−0.06	19.5	−0.10	0.595
End-diastolic length	7.06	−44.5	0.68	**0.009**	1.08	7.49	−0.16	0.460
LV resting diastolic function								
E/A ratio	8.79	−3.16	0.38	0.161	−1.76	19.4	−0.10	0.630
LV resting myocardial deformation								
Peak systolic longitudinal strain	1.80	45.6	0.56	**0.031**	0.58	28.3	0.23	0.238

**Bold** p values are statistically significant (p < 0.05). LV = left ventricle; *m* = the slope (unstandardized regression coefficient), *b* = the intercept, *r* = Pearson correlation values for bivariate correlations; other abbreviations as in Table 2.

## Discussion

This study demonstrated for the first time that preterm-born young adults had a significantly impaired LV systolic response to physical exercise stress. Structurally, echocardiography revealed that prematurity was associated with greater LV mass and lower LV volumes indexed for body size, as previously shown by CMR (4). At rest, EF remained fully preserved, but increasing exercise intensity elicited a decline in EF, resulting in an overall lower EF than term-born control subjects. Submaximal COR was also lower, and LV length and degree of prematurity were highly predictive of this adverse systolic response in preterm-born individuals.

### Potential mechanistic links between preterm birth and heart failure

Recent large-scale epidemiological data provided evidence that being born preterm increased the risk of early heart failure (8). In line with this, preterm experimental models in rats showed prematurity-related stress could elicit LV remodeling and impaired systolic function before blood pressure elevation. Moreover, these early cardiac alterations increased susceptibility to developing heart failure secondary to the insult of persistent hemodynamic overload induced by angiotensin II infusion 17, 18.

It is consequential that the systolic deficits we observed manifested under moderate intensity physical exercise and were clearly evident in this cohort of healthy, normotensive, preterm-born young adults, which indicated that, apart from subsequent pathology or insult, prematurity alone confers this systolic impairment and diminished myocardial functional reserve. Further decrements over time to this already marginalized reserve capacity in this normotensive population would bring peak achievable systolic function increasingly nearer to baseline requirements (19). Hypertensive individuals were excluded from this study to avoid potential confounding from altered hemodynamics, treatment with antihypertensive medications, or other underlying cardiovascular risk factors. Despite the independence of the changes in LV systolic function during exercise from blood pressure, exposure to sustained blood pressure elevation or hypertension might have a greater cardiovascular impact over time in preterm-born individuals due to this reduced myocardial reserve (19). These new findings of impaired systolic response to exercise in preterm–born adults might help elucidate the mechanisms linking preterm birth to increased heart failure risk.

Immediate postnatal developmental alterations appear to be critical for determining future cardiac risk and vulnerability. Even modest prematurity significantly affects cardiac development (3), which likely contributes to reduced cardiac resilience throughout childhood and into adulthood. In preterm birth, the abrupt, premature transition to the ex utero environment and early reversal of ventricular workloads disrupts normal cardiac development and is understood to produce long-term impacts on the myocardium. In explant experiments, hearts from piglets delivered preterm showed poor stress response marked by excessively reduced LV output when challenged with increased afterload; a hemodynamic challenge similar to physical exercise (20). Our new findings indicated these deficits likely persist through development and into adulthood. Furthermore, a late preterm sheep model showed that preterm lambs had increased myocardial collagen deposition and altered cardiomyocyte ploidy, which suggested an accelerated and potentially disrupted process of postnatal heart maturation, which might result in long-term cardiac vulnerability (21). Subsequent evidence from human studies indicated that typical cardiac ploidy not only supports cardiac development, but also represents a limited cardiac regenerative capacity from birth through adolescence 22, 23. Accordingly, in those born preterm, myocardial reserve deficits may combine with a further limited capacity for early life cardiac regeneration, leading to a compounding of vulnerabilities for future heart failure.

### LV structure and function, early life history, and cardiac risk in the preterm population

A previously reported CMR study of the LV in 102 preterm-born adults (mean gestational age 30.3 ± 2.5 weeks) versus 132 term-born control subjects identified a unique cardiac morphology in the preterm-born group, with lower LV length being a major anatomical feature (4). Although this present study showed a similar percentage difference in LV length in preterm offspring compared with term-born individuals, the slightly later mean gestational age of the preterm group (32.8 ± 3.2 weeks), smaller sample size, and increased variance of echocardiography versus CMR (particularly with apical views) accounted for the lack of statistical significance. Nevertheless, the correlation between LV length and exercise systolic response was only evident in the preterm-born group and might play a future role as a structural biomarker for risk in preterm-born offspring.

Interestingly, in those born preterm, exclusive human milk feeding in early post-natal development was shown to relate to greater LV length and a general shift toward normalized cardiac structure and function in adulthood (24). These and other findings might help direct future targeted intervention strategies. The growing population of preterm-born adults with increased cardiovascular disease burden 1, 25, 26, 27 necessitates clinical risk stratification and prevention guidelines that include, at a minimum, basic elements of birth and early life history.

### Study limitations

We designed YACHT as an observational study around a single, full-day study visit. Because the exercise stress testing occurred toward the end of the visit in order not to confound other measures, not all individuals were willing to continue with the submaximal exercise testing and the echocardiography stress testing component. Also, due to challenges with imaging quality, not all scans were of sufficient quality for analysis. Finally, the overall sample size was modest, with a lower percentage of men in the preterm cohort; therefore, p values were adjusted for sex when appropriate. Despite this, this study was sufficiently powered to make between-group comparisons for our primary outcome measure, LVEF, at rest, and at 40%, 60%, and 80% of maximal exercise capacity using echocardiography, and all scans were anonymized to avoid bias during analysis, including image quality assessment.

Due to the retrospective nature of the perinatal data collection, we did not have complete information on perinatal characteristics and complications. Future prospective studies might be able to address whether specific early life insults alter LV function. There was a wide gestational age range in our participants, with most of our preterm-born individuals born moderate to late preterm, which reflected the demographic characteristics of the general preterm population (28). Although this made our findings more relevant to a larger proportion of the population, larger studies will be needed to fully explore to what extent the severity of the LV systolic response to exercise is altered specifically in very and extreme preterm-born adults.

Resting echocardiography was performed per clinical standards with subjects scanned in the lateral decubitus position (12); however, upright cycle ergometry and treadmill are the most common clinical exercise stress modalities (29). We selected upright, seated cycle ergometry for CPET and stress echocardiography to align with clinical norms and to also minimize torso movement during scanning. Although all participants received standardized, per-protocol measurements, the differing posture could confound the direct comparisons of some resting echocardiography versus exercise echocardiography measures, such as stroke volume (30).

## Conclusions

Preterm-born young adults exhibited a significantly impaired LV functional response to physical exercise. This impairment was characterized by a lower exercise EF, which declined with increasing exercise intensity, as well as a reduced submaximal COR. Resting echocardiography showed a significant relationship between birth history and LV structure and function that was consistent with our previous CMR findings. Most notably, the novel finding of impaired exercise response offered insights that might help explain the recently verified relationship between preterm birth and increased risk of early heart failure. Because >10% of young adults worldwide are born preterm, there is an increasing need for further research into whether lifestyle and clinical interventions can beneficially modify cardiac morphology and function in this growing population of individuals.

Perspectives **COMPETENCY IN MEDICAL KNOWLEDGE:** Preterm birth is an independent risk factor for heart failure early in life. In addition to altered cardiac morphology, young adults delivered before term have impaired LV responses to exercise compared with term-born control subjects, which are evident as reduced augmentation of LV EF and submaximal myocardial functional reserve.

**TRANSLATIONAL OUTLOOK:** Further research is needed to determine whether lifestyle and clinical interventions can favorably influence cardiac morphology and function in individuals delivered prematurely.
